This article has been retracted.

# Fourier Transform Infrared Spectroscopy vibrational bands study of *Spinacia oleracea* and *Trigonella corniculata* under biochar amendment in naturally contaminated soil

**DOI:** 10.1371/journal.pone.0253390

**Published:** 2021-06-30

**Authors:** Uzma Younis, Ashfaq Ahmad Rahi, Subhan Danish, Muhammad Arif Ali, Niaz Ahmed, Rahul Datta, Shah Fahad, Jiri Holatko, Tereza Hammerschmiedt, Martin Brtnicky, Tayebeh Zarei, Alaa Baazeem, Ayman EL Sabagh, Bernard R. Glick

**Affiliations:** 1 Department of Botany, University of Central Punjab, Punjab, Pakistan; 2 Pesticide Quality Control Laboratory, Multan, Punjab, Pakistan; 3 Department of Soil Science, Faculty of Agricultural Sciences and Technology, Bahauddin Zakariya University, Multan, Pakistan; 4 Department of Geology and Pedology, Faculty of Forestry and Wood Technology, Mendel University in Brno, Brno, Czech Republic; 5 Department of Agronomy, The University of Haripur, Haripur, Pakistan; 6 Department of Agrochemistry, Soil Science, Microbiology and Plant Nutrition, Faculty of Agrisciences, Mendel University in Brno, Brno, Czech Republic; 7 Faculty of Chemistry, Institute of Chemistry and Technology of Environmental Protection, Brno University of Technology, Brno, Czech Republic; 8 Laboratory of Tropical and Mediterranean Symbioses, CIRAD, Mintpellier, France; 9 Department of Biology, College of Science, Taif University, Taif, Saudi Arabia; 10 Department of Agronomy, Faculty of Agriculture, Kafrelsheikh University, Kafr El-Shaikh, Egypt; 11 Department of Biology, University of Waterloo, Waterloo, ON, Canada; Harran Üniversitesi: Harran Universitesi, TURKEY

## Abstract

Fourier transform infrared spectroscopy (FTIR) spectroscopy detects functional groups such as vibrational bands like N-H, O-H, C-H, C = O (ester, amine, ketone, aldehyde), C = C, C = N (vibrational modes of a tetrapyrrole ring) and simply C = N. The FTIR of these bands is fundamental to the investigation of the effect of biochar (BC) treatment on structural changes in the chlorophyll molecules of both plants that were tested. For this, dried leaf of *Spinacia oleracia* (spinach) and *Trigonella corniculata* (fenugreek) were selected for FTIR spectral study of chlorophyll associated functional groups. The study’s primary goal was to investigate the silent features of infrared (IR) spectra of dried leave samples. The data obtained from the current study also shows that leaf chlorophyll can mask or suppress other molecules’ FITR bands, including proteins. In addition, the C = O bands with Mg and the C9 ketonic group of chlorophyll are observed as peaks at1600 (0%BC), 1650 (3%BC) and 1640, or near to1700 (5%BC) in spinach samples. In fenugreek, additional effects are observed in the FTIR spectra of chlorophyll at the major groups of C = C, C = O and C9 of the ketonic groups, and the vibrational bands are more evident at C-H and N-H of the tetrapyrrole ring. It is concluded that C-N bands are more visible in 5% BC treated spinach and fenugreek than in all other treatments. These types of spectra are useful in detecting changes or visibility of functional groups, which are very helpful in supporting biochemical data such as an increase in protein can be detected by more visibility of C-N bands in FTIR spectra.

## Introduction

Environmental pollution is a serious hazard for all living things on earth. Many diseases in living organisms are either caused or exacerbated by environmental pollutants [1]. Unfortunately, the growth of many vegetables includes the use of highly polluted water that contains high levels of one or more heavy metals such as cadmium (Cd), lead (Pb), arsenic (As) and mercury (Hg). These pollutants are taken up by plants and eventually negatively impact many metabolic processes like photosynthesis, respiration, transportation, and nitrogen metabolism [2–9]. These metals can critically affect photosynthesis by damaging the chlorophyll present within plant’s chloroplasts [10]. Two basic chlorophylls (chlorophyll a and chlorophyll b) are involved in photosynthesis light reaction. Any alteration to their structure can inhibit the whole photosynthesis process [11, 12]. To avoid the inhibition of photosynthesis by metals from the environment, it is possible to augment growing plants with BC to immobilize heavy metals [13–15]. Biochar contains specific structural sites for the immobilization of heavy metals. The surface adsorption of metals on the carbonized material decreases heavy metals’ mobility [10, 14, 16–22]. In this way, food quality is also improved through BC treatment [23–27].

The involvement of FTIR for observing changes in vibrational modes of functional groups is a unique and new technique. It describes changes in functional groups very clearly. Whereas, data values of any treatment on the basis of increase or decrease can predict and support the effect of functional groups [28]. The vibrational modes of plant pigment, especially chlorophyll is monitored using FTIR. The absorption peak at 1653cm^-1^ in aliphatic hydrocarbons [29, 30] has been assigned to C-9 of ketone oxygen coordinated to Magnesium, i.e., C = O →Mg. This interaction ultimately results in dimer formation, usually used to characterize chlorophyll’s infrared spectroscopy in non-polar solvents. The absorption peak characteristic of this aggregation is at ~1650 cm^-1^. Short-wavelength shoulders indicate the presence of high aggregates in aliphatic hydrocarbons [31]. The absorption peak at 1695 cm^-1^ reflects the free ketone carbonyl absorption and ester carbonyl absorption is found at 1735 cm^-1^; however, this is not differentiated from the 1650–1660 cm^-1^ aggregation peak [29, 32]. Similarly, the absorption peak at 1695 cm^-1^ is considered a consequence of a small amount of free carbonyl in the absorbing species [33, 34]. For this reason, the absorption peak at 1638 cm^-1^ is associated with the ring vibration ketone oxygen, which is hydrogen-bonded to the hydrated central Mg of another molecule of chlorophyll.

A water molecule coordinated with a central Mg of one chlorophyll molecule can also be arranged to make a hydrogen bond with the ketone oxygen at C-10 of the carbonyl group of a separate chlorophyll molecule [35]. This interaction establishes ester carbonyl interaction to show two peaks at 1743 and 1727 cm^-1^, respectively. Therefore, three peaks, i.e., chlorophyll monomer, chlorophyll dimer, and chlorophyll-water aggregate are observed at 1660, 1653 and 1638 cm^-1^, respectively. These are known as aggregation peaks, but their origin and importance are quite different [33, 34]. The formation of prominent wave numbers and vibrational modes of the major spectral region (I-V) between 1760 and 1500 cm^-1^ in the FTIR spectrum of chlorophyll photosystem II was elaborated in detail by Zamzam et al. [36], Hasting and Wang [37] and Segui et al. [38]. The investigation of the dimerization of photo chlorophyll pigments in non-polar solvents was described by Rasquin et al. [39]. According to Rasquin et al. [39], the IR (infrared) spectrum in the region of 1600–1800 cm^-1^ clearly shows the coordination of C-9 Ketone-oxygen of one chlorophyll molecule with the central Mg atom of another molecule of chlorophyll. Similarly, the OH stretching region’s infrared spectra provide essential data to evaluate the sample’s water content.

Thus, peaks in the FTIR spectrum of the plant leaves are largely due to chlorophyll and from some protein components because these are present in excess and mask the peaks of other components found in plant leaves. The current study aimed to explore the influence of different BC application rates on the growth of *Spinacia oleracea* and *Trigonella corniculata* in naturally polluted soil. A primary goal was to observe particular characteristics of leaf chlorophyll that include intensity variations of the prominent bands and also to look for additional bands. It is hypothesized that metal toxicity can induce changes in characteristic peaks of the chlorophyll molecule. These changes help detect or suggest the effect of any functional group like C-N, Mg and ketone-oxygen, etc, on protein, chlorophyll, and other biochemical attributes of the plant. Therefore, this type of FTIR study provides basic support for suggesting any functional group’s involvement in the quantity of biochemical attributes in response to any treatment.

## Materials and methods

### Soil and biochar

The pot experiment was performed at the Botanical Garden, Bahauddin Zakariya University, Multan, Pakistan, using a completely randomized design (CRD) on spinach (*S*. *oleracea*) and fenugreek (*T*. *corniculata*) with BC (0, 3, and 5%) in naturally contaminated soil with four replicates. Different BC levels were main, while *S*. *oleracea* and *T*. *corniculata* were subfactors. The naturally contaminated soil for the experiment was collected from the Agricultural fields of Bahauddin Zakariya University, which were previously irrigated with wastewater and had the following characteristics; pH 8.1, EC 3.00 dS/m, organic matter 0.76%, Cd 17 mg/kg, Ni 22 mg/kg and were described in our previously published work Younis et al. [28]. The safe limit for plant survival are: Cd = 0.2 μg g^-1^ (WHO/FAO 2007 [40]; European Union Standard 2006 [41]) and Ni = 1.5 μg g^-1^ (Indian Standard 2000 [42]). Pyrolysis of cotton sticks was carried out in a stainless-steel furnace especially designed to prepare BC from cotton sticks in a limited air supply. For this purpose, cotton sticks were collected from a cotton field and chopped into 5 mm pieces. Then pyrolysis was carried at 450°C for a period of two hours. After cooling, grinding of BC was done to 2 mm for utilization in the experiment. The BC has the following physicochemical properties; pH 9.5, EC 1.52 dS/m, N 1.12%, P 0.47% and K 1.6%, which our team already reported.

### Plant growth

The spinach and fenugreek plants were grown in clay pots (10-inch diameter and 12-inch depth) with a mixture of 5 kg of naturally contaminated soil and BC treatment. In each pot, 6 plants were grown and maintained. The experimental plants were irrigated regularly (50% water holding capacity of soil on a weight basis). After 45 days post germination, harvesting was done manually.

### Fourier transform infrared spectroscopy (FTIR)

The Fourier Transform Infrared Spectrophotometer (FTIR) of dried spinach and fenugreek leaves (composite sample of 4 replicates) was carried out to study the functional groups [32, 43]. It involves the following steps; 1. Preparation of potassium bromide (KBr) pellet. 2. Pressing of pellet at high pressure to make KBr disc. 3. KBr disc is ready for FTIR analysis. 4. Visualization of spectra by FTIR. To do this, 1.5–2.0 g of plant sample were gently mixed with 200 mg of solid KBr and ground to make a pellet. The standard device was used to make pellets under vacuum and pressure (75 kN cm^-2^) for 2–3 minutes (Fig 1). These pellets were then used for spectral analysis of functional groups by FTIR. The spectral resolution was 4 cm^-1^ with a 400–4000 cm^-1^ scanning range.

**Fig 1:** Procedure of Fourier Transform Infrared Spectroscopy usage for analysis of samples. Each subsection picture is showing the step involved in the analysis.

## Results and discussion

Fourier transform infrared spectrophotometer spectrum peaks were due to chlorophyll for most plant leaves, with a smaller contribution from some protein components. As in green leaves, a huge quantity of chlorophyll is present, which is more visible in color; that’s why chlorophyll can mask the other components. These components (chlorophyll) are found in abundance and mask the peaks of other components that are present in plant leaves. Therefore, we have focused on the characteristic peaks of chlorophyll molecules to assess the effects of various BC amounts on the growth of two different plants by treating the contaminated soil with BC. Studies that describe the bands originating from different groups (N-H, O-H, C-H, C = O, C = C and C = N) are characteristics of individual plant leaves (spinach and fenugreek) and show different intensities in BC treated and untreated plants. As the BC concentration was increased, characteristic peaks were increased in intensity, indicating the increased growth of plant chlorophyll and proteins. In contrast, untreated plants showed low intensities of these characteristic peaks of plant leaf components (Figs 2–5). This effect of BC was also observed by Younis et al. [28] during the characterization of BC by FTIR and biochemical attributes. They found that BC can increase nutrient uptake and water holding capacity of soil, which leads to better plant growth in the presence of contaminants.

**Fig 2:** FTIR spectrum of spinach leaves of a plant grown in naturally contaminated soil without BC [A]. FTIR spectrum of spinach leaves of a plant grown in naturally contaminated soil with 3% BC [B]. FTIR spectrum of spinach leaves of a plant grown in naturally contaminated soil with 5% BC [C].

**Fig 3:** FTIR spectrum of fenugreek leaves of a plant grown in naturally contaminated soil without BC [D]. FTIR spectrum of fenugreek leaves of a plant grown in naturally contaminated soil with 3% BC [E]. FTIR spectrum of fenugreek leaves of a plant grown in naturally contaminated soil with 5% BC [F].

**Fig 4:** Comparative FTIR spectra of spinach in naturally contaminated soil with 0, 3 and 5% BC.

**Fig 5:** Comparative FTIR spectra of fenugreek in naturally contaminated soil with 0, 3 and 5% BC.

Plants grown in soil treated with a higher level of BC show a better protein and chlorophyll profile, and this effect of BC is more prominent in spinach leaves than in fenugreek leaves. Nitrogenous peaks are more pronounced in plants grown with 5%BC as compared to untreated plants. Thus, BC (5%) trapped the heavy metals and prevented them from being taken up by the plant, which increased growth, a situation that is supported by the FTIR spectra of fenugreek and spinach. That is, chlorophyll and nitrogenous content are much higher in 5% BC treated plants as compared to untreated plants.

The understanding of the chlorophyll infrared spectra is based on the work of [44–46]. Carbonyl is most significant region in these spectra, where majority of ligand absorption bands are attained. These positions of ligand absorption are less or more independent of metal ion bonds to the tetrapyrrole ring center. C-H vibrations are observed at ~2852–2921 cm^-1^ (Table 1). This result agrees with the band assignments in the literature for these C-H stretching modes at 2925, 2960 and 2875 cm^-1^ [45, 47]. Ketone [C = O] C-9 band is reported to appear as two bands, i.e., at normal ketone absorption (~1700 and ~1650 cm^-1^) ketone oxygen coordination to magnesium (at 1740 and 1650 cm^-1^) (Figs 1 and 2). Bands assignable to C-O, C-C and C-N vibrations are also observed. C-N vibrations of the tetrapyrrole ring assigned at position 5 [45], 1350 cm^-1^, are observed at ~1330–1340 cm^-1^ in spinach and ~1350–1430 cm^-1^ in fenugreek (Table 1).

**Table 1:** Vibrational modes of functional groups in spinach and fenugreek in the presence of BC (0, 3and 5%) and naturally contaminated soil.

Functional Groups	N-Hcm^-1^	O-H cm^-1^	C-H cm^-1^	C = Ocm^-1^ Ester/Ketone/ aldehyde	C = Ccm^-1^	C = Ncm^-1^vibrations of the tetrapyrrole ring	C = Ncm^-1^
Peaks in literature [Silver stein and Webster [29, 32, 48]	~3600–3860	~3400–3500	~2800–2970	C = O with Mg at ~1650	~1560–1650	~1300–1350	~1050–1100
				C9 ketonic of chlorophyll at ~1700			
[A] Spinach o% BC	-	~3191	~2852–2921	~1600	~1595–1600	-	-
[B] Spinach 3% BC	-	~3000–3300	~2800–2911	~1650		-	-
[C] Spinach 5% BC	~3600–3800	~3000–3500	~2800–2900	~1640, ~1700	~1400–1420	~1330–1340	~1050
[D] Fenugreek 0% BC	-	~3200–3500	~2800–2900	~1652	-	~1350	~1018–1070
[E] Fenugreek 3%BC	-	~3200–3400	~2800–2900	~1627	~1458	~1363	~1050
[F] Fenugreek 5% BC	~3586	~3200–3500	~2800–2900	~1650	~1527	~1380–1430	~1050

The absorbance positions of different functional groups in both spinach and fenugreek treated with BC and naturally contaminated soils are shown in Table 1.

## Conclusions and future prospective

In conclusion, C = O with Mg and the C9 ketonic group of chlorophyll are observed at peaks of 1600 cm^-1^ (0% BC), 1650 cm^-1^ (3% BC) and 1640 cm^-1^ or near about 1700 cm^-1^ (5% BC) in spinach samples. In fenugreek, additional effects are noted in the FTIR spectra of chlorophyll at C = C, C = O and C9 of ketonic groups. The vibrational bands were more evident for the C-H and N-H bonds of the tetrapyrrole ring. However, the C-N bands are more visible in 5% BC treated spinach and fenugreek with all treatments. In the future, by studying FTIR spectra, we can easily describe the role of different functional groups in any biochemical attribute like chlorophyll, protein, ascorbic acid etc., of the plant. It’s also possible to illustrate the structural changes in the biochemical molecule.
